RETRACTED

# Diminished AdipoR1/APPL1 Interaction Mediates Reduced Cardioprotective Actions of Adiponectin against Myocardial Ischemia/Reperfusion Injury in Type-2 Diabetic Mice

**DOI:** 10.1155/2023/7441367

**Published:** 2023-02-20

**Authors:** Chao Ren, Wei Yi, Bo Jiang, Erhe Gao, Jiali Liang, Bo Zhang, Zhe Yang, Dezhi Zheng, Yong Zhang

**Affiliations:** ^1^Department of Cardiac Surgery, No. 960 Hospital of PLA, Jinan City, Shandong Province, China; ^2^Department of Cardiovascular surgery, Xijing Hospital, Air Force Military Medical University, Shaanxi, China; ^3^Department of Cardiac surgery, General Hospital of Ningxia Medical University, Ningxia Medical University, Ningxia, China; ^4^Center for Translational Medicine, Temple University, Pennsylvania, USA

## Abstract

**Background:**

Obesity-related diseases have important implications for the occurrence, severity, and outcome of ischemic heart disease. Patients with obesity, hyperlipidemia, and diabetes mellitus (metabolic syndrome) are at increased risk of heart attack with decreased plasma lipocalin levels, and lipocalin is negatively correlated with heart attack incidence. APPL1 is a signaling protein with multiple functional structural domains and plays an important role in the APN signaling pathway. There are two known subtypes of lipocalin membrane receptors, AdipoR1 and AdipoR2. AdioR1 is mainly distributed in skeletal muscle while AdipoR2 is mainly distributed in the liver.

**Objective:**

To clarify whether the AdipoR1-APPL1 signaling pathway mediates the effect of lipocalin in reducing myocardial ischemia/reperfusion injury and its mechanism will provide us with a new approach to treat myocardial ischemia/reperfusion injury using lipocalin as an intervention and therapeutic target.

**Methods:**

(1) Induction of hypoxia/reoxygenation in SD mammary rat cardiomyocytes to simulate myocardial ischemia/reperfusion; (2) downregulation of APPL1 expression in cardiomyocytes to observe the effect of lipocalin on myocardial ischemia/reperfusion and its mechanism of action.

**Results:**

(1) Primary mammary rat cardiomyocytes were isolated and cultured and induced to simulate MI/R by hypoxia/reoxygenation; (2) lipocalin inhibited H/R-induced apoptosis in cardiomyocytes; and (3) APN attenuated MI/R injury through AdipoR1-APPL1 and the possible mechanism.

**Conclusion:**

This study demonstrates for the first time that lipocalin can attenuate myocardial ischemia/reperfusion injury through the AdipoR1-APPL1 signaling pathway and that the reduction of AdipoR1/APPL1 interaction plays an important role in cardiac APN resistance to MI/R injury in diabetic mice.

## 1. Introduction

In recent years, the widespread use of arterial bypass surgery, thrombolytic therapy, percutaneous transluminal coronary angioplasty, cardiac surgery with cardiopulmonary bypass, and cardiopulmonary resuscitation has made it possible to restore blood flow to the ischemic heart in a short time, leading to recovery of damaged structures, cardiac function, and improved health [1–4].

RETRACTED

APN is an adipocytokine synthesized and secreted by white and brown adipose tissue [5]. APN has three functions. First, it is an important regulatory hormone that prevents insulin sensitivity and tissue inflammation [6]. APN acts directly on the liver, skeletal muscle, and blood vessels, increasing insulin sensitivity by modulating AMPK activity and also inhibiting vascular inflammatory responses [7, 8]. APN levels are further decreased, and the antagonistic effect of APN on TNF-*α* in turn inhibits APN synthesis [9, 10]. Furthermore, thiazolidinediones (which antagonize TNF-*α*) can increase APN secretion from adipocytes [11, 12]. APN also has atherosclerotic effects, and recent reports indicate that APN plays an important regulatory role in the development and progression of several cardiac diseases [13, 14].

APPL1 is a signaling protein with multiple functional structural domains [15]. Two subtypes of lipoalkali receptors are known, AdipoR1 and AdipoR2 [16, 17]. Numerous studies have shown that APN in skeletal muscle has a protective effect, mainly because it activates AMPK via APPL1 [18, 19]. Extensive recent experimental results have shown that the APPL1-AMPK signaling axis mediates the beneficial metabolic effects of lipocalin in the heart. In the myocardium, lipocalin can regulate myocardial glycolipid metabolism by activating downstream signaling molecules through the AdipoR1-APPL1 signaling pathway. The protective role of APPL1 in the early stages of myocardial ischemia/reperfusion has not been reported, and the possible involvement of APPL1-dependent signaling pathways is also unknown. Interactions with androgen receptor, epidermal growth factor (EGF) receptor, follicle-stimulating hormone receptor, and APN receptor have been reported. Several studies have shown that the interaction between APPL1 and AdipoR mediates the metabolic modulatory and endothelial protective effects of APN. However, whether the interaction between APPL1 and AdipoR1 (the major APN receptor in cardiomyocytes) mediates the cardioprotective effects of APN against MI/R disorders and, therefore, is involved in the mechanism of cardiac APN resistance in type-2 DM remains to be examined.

Lipocalin is a new target for the treatment of insulin suppression, type-2 diabetes, and metabolism-related diseases. The study of APPL1 may enhance our current understanding of the lipocalin and insulin signaling pathways. Furthermore, it is indispensable for our study of the lipocalin signaling pathway and the insulin-sensitizing effects of lipocalin. Although the study of APPL1 has been progressed in some fields, its role in lipocalin-mediated myocardial ischemia/reperfusion injury is limited. Does APPL1 participate in the role of lipocalin in reducing myocardial ischemia/reperfusion injury? What are the molecular mechanisms through which APPL1 mediates the protection of lipocalin against ischemia/reperfusion myocardium? Therefore, we used this experiment to demonstrate the role of APPL1 in the protection of myocardial ischemia/reperfusion by lipocalin. This study will provide new targets for more effective clinical treatment of coronary artery disease and ischemic heart disease.

RETRACTED

## 2. Materials and Methods

### 2.1. Experimental Protocols

Forty-eight hours after RNAi injection, mice were anesthetized with 2% isoflurane and reperfused through an incision on the left side of the chest to induce a myocardial infarction (MI). Twenty minutes after MI, mice were randomly injected with APN (2 *μ*g/g) as vehicle or globule. At 30 min after infarction, the soluble compound was released, and the myocardium was resuscitated for 3 to 24 h (to determine cardiac function and infarct size). Control mice were operated sham, but the suture under the left coronary artery was not tightened.

### 2.2. Western Blot Analysis

The tissue was obtained from the MI mice 3 hours after reperfusion. The expressions of various proteins (APPL1, P-AMPK, AMPK, P-ACC, ACC, iNOS, and Caspase-3) were detected by Western blot as we previously described.

### 2.3. Neonatal Rat Primary Cardiomyocyte Culture

1. Preparation and dilution: prepare 100 ml of double antibody (add 5 ml saline to 5 ml streptomycin, shake well, then add 5 ml saline to the penicillin vial to dissolve, transfer all 5 ml to 95 ml saline, and divide into 10 vials). Prepare 100 ml DMEM culture solution containing 15% fetal bovine serum (85 ml DMEM, 15 ml fetal bovine serum, and 1 ml double antibody), and prepare 10 ml 0.1% collagenase I (10 mg collagenase I dissolved in 10 ml PBS). The solution is usually prepared in advance and filtered through a 0.22 pore filter
2. Irradiation with UV light for 20-30 min (2 culture flasks, 2 15 ml centrifuge tubes, and 4 lunch boxes were placed on the UV table)
3. SD mice immersed in 75% alcohol (5~10 min)
4. Add two drops of medium (DMEM + serum + double antibodies) to one vial of medium, and leave the other vial of medium undisturbed and screwed to one side of the ultrathin table (note: this step can be performed with a 50 ml pipette)
5. Take another dropper with a straight tip, rinse it, insert PBS, then remove the round container set, and add the appropriate amount of PBS
6. Take the heart. Six milk mice can be sewn sequentially onto a plastic foam plate using a broad-headed needle, and then open the chest sequentially using scissors to reveal the heart. Take another knife and forceps, lift the heart, cut it out, place it in a round dish with prechilled PBS, rinse the heart 2 times with PBS, and cut it out (1 mm × 1 mm × 1 mm)
7. Remove the drop and aspirate the PBS; then take the penicillin vial and transfer the excised myocardial tissue into the penicillin vial into the penicillin vial. Add 2 drops of collagenase I (approximately 3 ml) to the penicillin vial with dropper. After 10 minutes, add collagenase I (approximately 3 ml) to the dropper vial, close tightly, and leave for 10 minutes in a water bath at 37°C. After 10 minutes, add the digestion solution to the centrifuge tube with DMEM to complete the digestion
8. Centrifugation (room temperature, 1000 rpm, 10 min/time)
9. Through a 200-mesh sieve, after centrifugation, discard the supernatant, and use the medium in a third tube to resuspend the cells. After centrifugation, discard the supernatant, resuspend the cell pellet with the medium in the third centrifuge tube, take another set of round dishes, pass the cell suspension through a 200-mesh sieve, and then collect the sieved cells

RETRACTED

### 2.4. Induced Cardiomyocyte Hypoxia/Reoxygenation (H/R) Simulating Myocardial Ischemia/Reperfusion (MI/R)

The culture medium was replaced with ischemic blood (sodium hypodisulfate 0.75, KCl 12, lactate 20 mmol/L, pH 6.5). Three different anoxia/reoxygenation times were selected for experimental observation, which were sequentially set to incubate in anoxic incubator at 37°C: 6 h, 12 h, and 24 h. Then, the normal incubation medium was replaced and incubated in 5% CO2 incubator at 37°C for 3 h, 6 h, and 12 h, respectively, for testing.

## 3. Results

### 3.1. The AdipoR1-APPL1 Interaction Was Decreased in HD Mice

As an important regulator of APN metabolic signaling, APPL1 binds to AdipoR1 and mediates AMPK activation in the axon. We and others have shown that the cardioprotective effects of APN are attenuated in a diabetic state characterized by APN resistance. And we have found that the AMPK pathway and the antinitrogen/oxidant pathway are at least partially inhibited. However, we did not investigate whether the AdipoR1-APPL1 interaction is reduced in mice with type-2 diabetes. To determine the mechanism of APN resistance, we first detected the AdipoR1-APPL1 interaction by coimmunoprecipitation in HD-induced type-2 diabetic mouse hearts. Compared with HD hearts, neither AdipoR1 nor APPL1 expression was significantly altered in the protein level in HD mouse hearts. However, the coimmunoprecipitation of AdipoR1 and APPL1 in HD hearts was dramatically reduced (51.6%), suggesting that the interaction between APPL1 and AdipoR1 was greatly reduced in HD mice (Figure 1).

RETRACTED

### 3.2. Knockdown APPL1 Protein Expression by Infecting Stealth RNAi In Vivo

To investigate the role of the AdiopR1-APPL1 interaction in the in vivo regulation of APN cardioprotection, we deleted the APPL1 adaptor protein by intramyocardial injection of APPL1 stealth siRNA, as previously described. As shown in Figure 2 compared with scrambled siRNA injection, APPL1 protein levels in APPL1 knockout hearts were reduced by approximately 73.6%, as determined by Western blotting.

### 3.3. Cardioprotective Effect of APN Was Abolished in APPL1 Knockdown Mice

Having successful knockdown APPL1 expression by infecting APPL1 specific stealth RNAi, we determined to confirm whether the cardioprotective effect of APN would be affected.  Figure 3 shows that the cardioprotective effect of APN to MI/R injury was partially abolished on the APPL1 knockdown mice. Specifically, without the administration of APN, knockdown APPL1 before MI/R has no statistical significant difference from the group with scramble siRNA. The conclusion above can also be seen from the result of echocardiography (Figure 3(b)). These results confirmed that APPL1 is an important molecule in APN-mediated cardioprotection. Since AdipoR1-APPL1 interaction was reduced in HD mice, the cardioprotective effect of APN was diminished in APPL1 knockdown mice, and we propose that reduced AdipoR1-APPL1 interaction is the mechanism of APN resistance in type-2 DM.

### 3.4. Inhibition of APPL1 Expression Blocked APN's Phosphorylation of AMPK-ACC Axis

Previous studies have shown that APN stimulates AMPK/ACC phosphorylation [11]. To determine the mechanisms responsible for the APN-induced loss of cardiopulmonary protection in APPL1 knockout mice, we first assessed the phosphorylation stimulated by AMPK and ACC. Compared with controls, phosphorylation of AMPK or ACC was increased in all MI/R-treated groups. Phosphorylation of AMPK and ACC was significantly increased after MI/R, but there was no statistically significant difference between MI/R groups for APPL1 or scramble siRNA (Figures 4(a) and 4(b)). Compared with controls, administration of gAPN (with siRNA bracketed siRNA) further increased the phosphorylation of AMPK and ACC. In addition, gAPN treatment partially reduced phosphorylation of AMPK and ACC in APPL1 knockout hearts (Figures 4(a) and 4(b)), indicating that APPL1 is important for the APN-mediated AMPK signaling pathway.

RETRACTED

### 3.5. Cardiac Specific Injection of APPL1 Stealth RNAi Blunted Antinitrative and Antiapoptotic Effects of APN

As an overproduction of peroxynitrite, inducible nitric oxide synthase (iNOS) indicates a lack of source. As shown in Figure 5(a), APPL1 deficiency treatment of APPL1 knockdown hearts with gAPN increased MI/R-induced iNOS expression to levels comparable to those observed in normal hearts with APPL1 with gAPN, suggesting that APPL1 knockdown expression may impair the antinitrative effect of APN.

Our aforementioned experimental results showed that APPL1 is required for both AMPK-dependent and AMPK-independent APN signaling. We further evaluated the antiapoptotic effect of APN. Myocardial apoptosis was determined by the caspase-3 expression. As shown in the figure, no significant difference in caspase-3 expression was observed between normal hearts and APPL1 beating hearts. Treatment of wild-type mice as well as APPL1 knockdown mice with gAPN significantly suppressed caspase-3 expression. However, the absolute level of caspase-3 expression remained higher in gAPN-treated APPL1 knockdown hearts than in normal APPL1-treated hearts (Figure 5(b)). Together with the data presented in Figure 5(b), the results demonstrated that the MI/R-induced decrease in caspase-3 expression under gAPN was partially abolished when APPL1 was knocked down, indicating that APPL1 acts on the antiapoptotic effects of APN.

Our previous studies have demonstrated that HD impaired APN-induced AMPK-ACC activation and antinitrative protection [2]. Moreover, blunted antiapoptotic effects of APN in APPL1 knockdown mice indirectly indicating the effect of APPL1 in HD induced type-2 diabetic mice. Having determined that the AdipoR1-APPL1 interaction was reduced in HD mice, demonstrating that reduced AdipoR1-APPL1 interaction is the molecular mechanism of the cardiac APN resistance in HD induced type-2 DM.

### 3.6. APPL1 Stealth RNAi Blunted Anti-Cell Death Action of gAPN in Neonatal Cardiomyocyte

Yet in vivo experimental results, we have demonstrated that the interaction of AdipoR1 and APPL1 was decreased in HD-induced DM and the effect of APPL1 in APN preventing MI/R injury in cardiac. To obtain more evidence to support our plan, an additional study was performed by cultured neonatal rat primary cardiomyocytes. Cardiomyocytes were treated with APPL1 siRNA or scrambled siRNA and hypoxia/reoxygenation to simulate ischemia/reperfusion (SI/R) in the presence or absence of APN. First, the effect of APPL1 siRNA in cardiomyocytes was assessed by APPL1 expression. The APPL1 protein level was decreased by approximately 50% in the cardiomyocyte with APPL1 siRNA, which is a little higher than the results in vivo (Figure 6(a)). Since the APPL1 expression was successfully knockdown, the effect of gAPN on SI/R-induced cell death (Figure 6(b)) demonstrates that knockdown APPL1 is capable of blocking APN-induced cardiomyocyte anti-cell death.

RETRACTED

### 3.7. Inhibition of APPL1 Expression Partially Mimicked APN Resistance in HGHL-Treated Neonatal Cardiomyocyte

Our aforementioned in vivo experiment results have demonstrated that AdipoR1-APPL1 interaction is the molecular mechanism of the cardiac APN resistance in HD-induced type-2 DM. To further confirm it in vitro, HGHL cardiomyocytes were performed to simulate induction of type-2 DM as described previously to see APN resistance. As shown in Figure 7, cardiomyocyte apoptosis was determined by TUNEL. However, the effect of APN is partially abolished on cardiomyocyte cultured with either HGHL or APPL1 siRNA, which indicates that inhibition of APPL1 expression partially mimicked APN resistance in HGHL-treated neonatal cardiomyocyte. From Figure 7, cardiomyocyte culture in HGHL showed significantly increased TUNEL-positive cells, as provided from our previous study: type-2 diabetics manifested greater MI/R injury suffering.

## 4. Discussion

Myocardial ischaemia/reperfusion is an important risk factor for heart failure, and many studies have been proposed to identify the main mechanisms leading to cardiac remodelling. In particular, apoptosis-induced cardiomyocyte depletion is an important factor contributing to the progressive worsening of left ventricular hypertrophy, which may eventually lead to end-stage cardiomyopathy. With the development of research, adipocytokines are considered important factors regulating pathophysiological changes in heart failure and are strongly associated with the occurrence, progression, and prognosis of cardiovascular disease. The role of lipocalin in reducing myocardial apoptosis has been clearly demonstrated in numerous studies, effectively reducing acute myocardial ischaemia/reperfusion injury as well as apoptosis induced by chronic coronary syndrome. Recently, lipocalin has been shown to reduce cardiomyocyte apoptosis via AMPK-dependent signaling pathways and to reduce tumour necrosis factor (TNF-*α*) production via COX-2/PGE2-dependent molecular signaling mechanisms; lipocalin also exerts these protective effects by reducing oxidative/nitrosative stress and Akt activation. However, the exact mechanism remains to be elucidated.

Lipocalin exerts its physiological effects by binding to lipocalin receptors on the cell membrane and regulating several metabolic processes. Studies [8] using a yeast two-hybrid approach identified the first protein, APPL1, which binds directly to lipocalin receptors expressed in insulin-sensitive tissues such as muscle, liver, and adipose tissue and contributes to lipocalin signaling. APPL1 has several functional structural domains, of which the PTB structural domain binds to lipocalin receptor I (AdipoR1) and plays an important role in the lipocalin signaling pathway. Studies [1] have shown that in skeletal muscle, lipocalin activates AMPK via an APPL1/LKB1-dependent signaling pathway. In turn, lipocalin stimulates APPL1 interaction with AdipoR1. Increasing mutant APPL1 levels without the ability to bind AdipoR1 or inhibiting APPL1 with siRNA significantly attenuated lipocalin-induced AMPK, p38MAPK and ACC phosphorylation, and fatty acid oxidation, suggesting that APPL1 plays an important role in lipocalin-regulated lipid metabolism in skeletal muscle cells; APN promotes LKB1, mainly through APPL1/LKB1 APN that promotes the intracytoplasmic localisation of LKB1, which ultimately leads to AMPK activation, mainly through APPL1/LKB1-dependent signaling pathways.

RETRACTED

Studies [5] on the effects of lipocalin on myocardial metabolism using primary cardiomyocyte culture and isolated cardiac perfusate showed that lipocalin increases the interaction between AdipoR1 and APPL1, and finally, APPL1 binds to AMPK and is phosphorylated to inhibit ACC and increase fatty acid oxidation; using siRNA to decrease APPL1 expression in rat mammary cardiomyocytes, lipocalin function was inhibited. These experiments confirmed that APPL1 plays an important role in lipocalin-mediated myocardial metabolism. It is unclear whether lipocalin-stimulated AdipoR1 binding to APPL1 is involved in the role of lipocalin in reducing myocardial ischaemia/reperfusion.

In this study, we examined the important role of APPL1 in reducing myocardial injury during ischemia/reperfusion by isolating and culturing primary SD mouse cardiomyocytes and creating a hypoxia/reoxygenation model to simulate myocardial injury during ischemia/reperfusion. Primary isolation and culture of milk rat SD cardiomyocytes were used to simulate ischemia/reperfusion injury by hypoxia/reoxygenation of cells, and it was found that hypoxia/reoxygenation can significantly increase cardiomyocyte apoptosis and that after 12 h of hypoxia, a large number of cardiomyocytes undergo apoptosis, but that apoptosis is significantly reduced after lipocalin treatment, suggesting that lipocalin may play a cardioprotective role in I/RI. In addition, APPL1 expression in cardiomyocytes was significantly higher in the lipocalin-treated group compared with the control and H/R groups. To further test the role of APPL1 in the protective mechanism of apoptotic damage to cardiomyocytes by lipocalin, we found that the apoptosis index of cardiomyocytes was significantly increased after the inhibition of APPL1 expression in cardiomyocytes by RNA interference, which blocked the antiapoptotic effect of lipocalin on cardiomyocytes during I/RI, confirming that lipocalin inhibition of I/RI-induced cardiomyocyte apoptosis was associated with APPL1. In addition, we examined cell survival by MTT assay, which was significantly higher after lipocalin treatment compared with the H/R group and significantly lower in the interferon group compared with the H/R+g Ad group after inhibition of APPL1 expression. The expression levels of p-AMPK, p-e NOS and iNOS were determined by Western blot, and it was found that the expression levels of p-AMPK, p-e NOS, and iNOS were significantly reduced and increased after APPL1 inhibition. It is suggested that lipocalin may reduce myocardial injury during ischemia/reperfusion via the AdipoR1-APPL1-AMPK signaling pathway and that the AdipoR1-APPL1 signaling axis is also involved in the antioxidant/nitrosative stress effect of lipocalin.

RETRACTED

## Figures and Tables

**Figure 1:** Interaction of AdipoR1 and APPL1 was blunted in HD induced type-2 diabetic heart in mice. (a) Coimmunoprecipitation. The interaction of AdipoR1 and APPL1 was detected in ND or HD mice. ^∗∗^*P* < 0.01 vs. ND mice.

**Figure 2:** Interaction of AdipoR1 and APPL1 was blunted in HD induced type-2 diabetic heart in mice. Western blot analysis for APPL1. APPL1 expression was compared for groups with or without APPL1 siRNA. ^∗∗^*P* < 0.01 vs. the same treatment group without APPL1 siRNA.

**Figure 3:** Cardiac specific injection of APPL1 stealth RNAi blunted cardioprotective actions of APN against MI/R injury. (a) Myocardial infarct size. Determined by Evans blue/TTC double staining. (b) Cardiac function. Determined by echocardiography. ^∗∗^*P* < 0.01 vs. the same treatment group without APPL1 siRNA. ^&^*P* < 0.05; ^&&^*P* < 0.01 vs. the same treatment group without gAPN.

**Figure 4:** Inhibition of APPL1 expression blocked gAPN's phosphorylation of the AMPK-ACC axis.

**Figure 5:** Cardiac specific injection of APPL1 stealth RNAi blunted antinitrative and antiapoptotic effects of APN. (a) iNOS expression by representative Western blots. (b) Caspase-3 expression by representative Western blots. ^∗^*P* < 0.05 vs. the same treatment group without APPL1 siRNA. ^&^*P* < 0.05; ^&&^*P* < 0.01 vs. the same treatment group without gAPN.

**Figure 6:** APPL1 stealth RNAi blunted anti-cell death action of gAPN in neonatal cardiomyocytes. (a) Western blot analysis for APPL1. APPL1 expression was compared for groups with or without APPL1 siRNA. (b) LDH release. Cell death was determined by detection of LDH release. ^∗∗^*P* < 0.01 vs. the same treatment group without APPL1 siRNA. ^&^*P* < 0.05; ^&&^*P* < 0.01 vs. the same treatment group without gAPN.

RETRACTED

**Figure 7:** Inhibition of APPL1 expression partially mimicked APN resistance in HGHL-treated neonatal cardiomyocyte. Cardiomyocyte apoptosis was determined by TUNEL staining. ^∗^*P* < 0.05; ^∗∗^*P* < 0.01 vs. the same treatment group without gAPN. ^&&^*P* < 0.01 vs. the same treatment group without HGHL (with scramble siRNA).

## Data Availability

The experimental data used to support the findings of this study are available from the corresponding author upon request.
